This article has been retracted.

# Development of Novel Bio-mulberry-Reinforced Polyacrylonitrile (PAN) Fibre Organic Brake Friction Composite Materials

**DOI:** 10.1155/2022/6426763

**Published:** 2022-07-11

**Authors:** Naresh Kumar, L. Natrayan, G. Kasirajan, S. Kaliappan, M. D. Raj Kamal, Pravin P. Patil, Muse Degefe Chewaka

**Affiliations:** ^1^Mechanical Engineering Department, Green Hills Engineering College, Solan 173229, India; ^2^Department of Mechanical Engineering, Saveetha School of Engineering, SIMATS, Chennai 602105, Tamil Nadu, India; ^3^Department of Mechanical Engineering, St. Joseph's College of Engineering, Chennai 600119, Tamil Nadu, India; ^4^Department of Mechanical Engineering, Velammal Institute of Technology, Chennai 601204, Tamil Nadu, India; ^5^Department of Mechanical Engineering, Graphic Era Deemed to be University, Dehradun 248002, Uttarakhand, India; ^6^Department of Mechanical Engineering, Ambo Institute of Technology–19, Ambo University, Ambo, Ethiopia

## Abstract

Natural fibre reinforcement is used in important sectors such as medical, aerospace, automobile, and many other fields. Many articles have reported that natural fibre has the potential to replace synthetic fibres. Natural fibre reinforcement has given good results as a brake friction material. It has already been proven that asbestos causes lung cancer and mesothelioma in brakes. Many people died from the effects of asbestos. According to the World Health Organization's trending brake report, this material leads to serious health issues. This work is going on for the replacement of these materials. Mulberry fibre is a unique material, and PAN fibre is combined with mulberry fibre and used as a brake reinforcement material to replace Kevlar fibre. The brake pads were fabricated with the various wt% of mulberry fibres and PAN fibre [3–12%] with an equal ratio and aramid fibre [3–6%] in the hydraulic hind brake moulding machine. The mechanical, chemical, physical, tribological, and thermal properties were evaluated. MF-2 [6 wt%] mulberry-PAN-fibre-based brake pad composites have shown better results for ultimate shear strength and proof stress, tensile strength, compressive strength, and impact energy.

## 1. Introduction

Synthetic fibres are replaced by organic fibres in many functions day by day. It has been investigated that there are many environmental issues with the trending brake friction materials. Natural fibres have been used by humans for many years [1]. These organic fibres are commonly used as carpets, ropes, clothes, interior applications, etc. Nowadays, these organic fibres are used to substitute synthetic fibres (reinforcement of polymer composites) [2]. Previous reports and studies show that asbestos used in various applications leads to the deaths of too many people. The use of asbestos started by keeping its advantage of excellent braking properties. However, further research has found that it leads to various kinds of cancers and causes serious lung disease [3]. After several environmental organizations raised the issue with the government, the use of asbestos was prohibited. Many researchers suggested replaceable materials, which could be a better alternative to asbestos [4]. Aramid is utilized in brake pads as a reinforced material today [5]. This reinforced material also has limitations, such as a lower recycling rate, high cost, and environmental toxicity [6]. Many articles have shown the serious harmful effect of aramid on human health [7]. Natural fibres as an alternative are light in weight and easy to shape, cheaper in cost, eco-friendly to the environment, and biodegradable. It also has good tensile strength and high specific strength [8]. The applications of natural fibres include bike helmets, automobile parts, and bulletproof materials [9]. Apart from having several advantages, it also has disadvantages like higher moisture absorption. But as per information from different articles, the properties such as porosity, tension, wetting, and adhesion strength of the surface can be modified by performing different chemical treatments [10]. Based on the classical filtration theory, filtration using fibrous materials has been divided into five mechanisms for trapping particulate matter: interception, Brownian diffusion, inertial impaction, and electrostatic gravitational effect [11]. The particulate matter closer to the fibres generally deviates from the gas flow streamlines as the filtration occurs. This deviation affects the performance of the fibrous material as a filter media. The deviation occurs via the following five mechanisms. The interception of PM occurs when the van der Waals interaction results in contacting the surface of the fibrous membrane, assuming that PM follows a flow line and no deviation occurs [12]. PM capture usually occurs through the interception mechanism for particle sizes of 0.1 to 1 *μ*m. As the particle size decreases, Brownian motion is favoured. The collision of PM with fibres results in the deposition. PM deviates randomly from its original flow during the Brownian motion and gets captured when this deviation is larger enough to impact the fibre and the PM [13]. Brownian diffusion is generally exhibited for particles smaller than 0.1 *μ*m. High filtration efficiency and lower pressure drop are the essential properties of an efficient electrospun nanofibrous membrane to filtrate PM from the atmosphere [14]. For higher filtration efficiency, it is necessary to have smaller fibre diameters. The fibrous materials' smaller pores are efficient in completely removing particles larger than them due to the sieving effect. Thus, the electrospun nanofibrous materials with smaller pore sizes efficiently remove ultrafine particles [15].

MWCNTs have been successfully employed in the positive sulfur electrode for many benefits. It showed that sulfur-impregnated disordered CNTs obtained by a vapour infusion method were capable of trapping polysulfide species. CNFs have morphological features similar to CNTs except for the central core. Moreover, their high conductivity and structural strength make them attractive constituents in sulfur carbon composite electrodes. They can also form network structures that can suppress the agglomeration of S/Li_2_S on the electrode [16]. A composite electrode with a 3-D network of CNF clusters was shown to suppress active material accumulation. High initial capacities exhibited by sulfur CNF composites are attributed to enhanced conductivity and immobilization of active sulfur in the porous structure of CNFs [17]. Engineered hierarchically porous carbons such as CMK-3 offer high sulfur utilization due to the complete redox reaction within the confined nanosized pores. These carbons have an architecture in which the micropores encapsulate the active material. The macropores serve as excellent percolation paths for the electrolyte. Such hierarchically porous carbons act as electronic conduits and a stockroom for the active material. The excess usage of fertilizers and pesticides on crops is the major source of chemical pollution. The untreated industrial and domestic effluents are also significant sources of water pollution [18]. The groundwater contamination through the effluents from agrochemical industries creates huge health problems. Heavy metal ions enter the human body through habits like drinking and eating. In recent years the government has made strict laws for the safe discharge of these toxic metal ions [19].

Mulberry fibre is found in the resign of the Himalayans and mostly in the northern zone of India. It is a very fast-growing plant, and its stems are used to collect the fibres. The mechanical properties of mulberry fibre were good in some articles [20]. PAN fibre is used in hot gas filtration systems, concrete reinforcement, sweater and socks manufacturing, and other applications due to its good mechanical properties [21]. Some natural fibres have been used as reinforcement materials, even though PAN has good frictional properties. A novel of this research work is to develop the novel bio-mulberry-reinforced polyacrylonitrile (PAN)/aramid organic fibre brake friction composite materials using hydraulic hind brake moulding machine. Fabricated organic composite's mechanical, chemical, physical, tribological, and thermal properties were evaluated.

## 2. Materials and Methods

### 2.1. Materials and Composite Fabrication

Mulberry fibres were collected using the traditional method. Mulberry stems were obtained from the tree of mulberry, and the leaves were eliminated [22]. Then, mulberry stems were put into the water for 4 weeks, and after that, the fibre was extracted from the steams. The extracted fibre was then washed with deionized water and put in the sunlight for two days. The collected fibre was treated with sodium hydroxide [NaOH] by immersing it for 24 hours to eliminate any possible impurities. The extracted fibre was cut into 1–5-mm pieces [23].  Figure 1 shows the PAN fibre, (b) raw material of mulberry fibre, C) developed brake pads of mulberry-PAN fibre. PAN fibre and other brake materials were available in Allied Nippon, Ghaziabad [24]. Then, these small pieces were mixed with other materials (aluminum oxide, phenolic resin, barium sulphate [BaSO_4_], potassium titanate, graphite, and vermiculite) used for the development of brake pads [25]. The procedure and composition are shown in Tables 1 and 2.

### 2.2. Characterization of Physico-Mechanical and Thermal Properties

The automobile used for this test sample was dipped for two days to measure the porosity [26]. A Glun Digital pocket scale was utilized for the measurement of density. The apparatus used to find the uncured resin is called “acetone extraction” [27]. The common way to determine the water absorption by new samples is to put them into the water for one day [ASTMD570-98 standard]. Mechanical properties were found with the universal testing machine [28]. An impact test was performed with the help of a pendulum impact testing machine. The flexural test was performed with the help of an automatic flexural testing machine [29]. The new hybrid specimen was heated up at 700°C to determine the ash percentage [30]. The sample size was taken 60 × 20 × 10 mm for mechanical properties and friction tests; the size was taken 40 × 40 × 10 mm [31].

### 2.3. Thermo-Gravimetric Analysis

TGA was evaluated on TA-60WS [heat rate = 10°C/min, temperature = 40–800°C, Sample Size = 10 mg] in an nitrogen atmosphere [flow rate of nitrogen [N_2_] = 45 ml/min]. The experiment was performed at Allied Nippon, Ghaziabad. The oxidation index (OI) was calculated based on the weight of carbonaceous char (CR) [32].

### 2.4. Testing of Tri-Biological Characteristics of Developed Composites

A chase machine was used to investigate the tribological properties of the manufactured new samples [33]. This test has investigated the fade cycle, recovery cycle, fade percentage, wear, stability, recovery percentage, and variability [34]. The first fad and recovery cycle started with the burnishing of the sample at 350 rpm. The starting condition was maintained (L [load] = 400 N, *T* [temperature] = 95°C, and *t* [time taken] = 25). The contact between the rim and samples was noticed at 90%. For the first and second cycles, speed and load were maintained at 400 rpm and 700 N, respectively. The regulator maintained the temperature [95–300°C]. The reading was taken at various temperatures for the first fade (245°C, 195°C, 145°C, and 95°C). Other conditions were maintained for second fade cycles (295°C, 245°C, 195°C, 145°C], and frictional properties were recorded after 50°C. The various parameters have been evaluated at the end of the test. (A) Fade: fade is known as heat generated by friction between the brake surfaces [35]. The brake efficiency decreased with the higher value of fade. It is undesirable for frequently breaking or intermittent breaking [stop and go city drive conditions. (B) After releasing the brakes, the brake lining gets cool, and the value of *µ* reaches its original (friction) level, which is called recovery. (C) %-Fade = *µ*p-*µ*F/*µ*p × 100, D) %-Recovery = *µ*R/*µ*P × 100; consider 100–120% for good brake pad friction composites. (E) Stability coefficient (*Sμ*) = *µ*_P_/*µ*max; it should be as high as possible. (F) Variability coefficient (*Vμ*) = *µ*min/*µ*max; it should be as least as possible [36]. (G) Wear = W1–W2; W1 is the starting weight of the composite samples (before test) and W2 is the ending weight of the composite samples (after test). (H) Coefficient of performance (µP): it has been seen that, at the high temperatures (more than 100°C), the value of *µ*_*P*_ has remained average COF for all cycles (recovery and fade). The picture of the chase machine used for the tribological test is shown in Figure 2.

## 3. Results and Discussion

### 3.1. Characterizations of Chemical, Physical, Mechanical, and Tri-Biological of Mulberry Fibre and PAN Fibre/Aramid Fibre Composites

The compressive strength was found to be the highest for MF-2 = 176.7 MPa and KV-2 = 167.5 Mpa and lowest for MF-4 = 140.6 and KV-1 = 162.3 Mpa. The observation was that at 6% mulberry fibre and PAN fibre, wall fibre composition produces the uniform matrix [37]. The maximum shear strength values were MF-2 = 2520 kgf and KV-1 = 1890 kgf. One possible reason might be the increased percentage [3–6%] of mulberry fibre and PAN fibre, which must have behaved as the binder, but upon increasing it more [9–12%], the fibre composite has shown an uninformed matrix. Failure strain was found to be the lowest for MF-1 and KV-1 [1.48 and 1.20] and the highest for MF-4 and KV-2 [1.69 and 1.24]. Proof stress was significantly higher for composites MF-2 and KV-1 [3.6% and 3.4%) and lower for MF-1 and KV-2 [2.75% and 2.90%]. As shown in Table 3, MF-1 and KV-1 composites show the highest flexural strength values and flexural modulus [38]. The porosity of the polymer composites increased as the percentage of mulberry fibre-PAN fibre and aramid fibre was increased [mulberry fibre-PAN fibre = 3.4–4.05% and aramid = 3.25–3.32%] in the polymer matrix. It occurred due to improper mixing of the constituents in the polymer matrix [39]. It was noticed that the ash content decreased with the increase in the weight percentage of mulberry fibre (PAN fibre and aramid fibre) [40].

In the new devolved composites, the highest value of the ash content was observed in a 3 wt.% proportion [mulberry fibre, PAN fibre = 74.75%, and aramid = 75.30%]. The water absorption capacity of the polymer was increased with the increase in the mulberry fibre-PAN fibre and aramid content [mulberry fibre-PAN fibre = 2.95–3.90% and aramid = 2.70–2.81%]. Water absorption was found to be lower [mulberry fibres-PAN fibre = 1.77% and aramid = 1.70%] for MF-1 and KV-1, and the water absorption capacity of the polymer matrix was found to be maximum [mulberry fibre-PAN fibre = 3.90% and aramid = 3.30%] for MF-4 and KV-2. The compressibility was observed to be low [mulberry fibre-PAN fibre = 1.40% and aramid = 1.25%] for MF-1 and KV-1, and for a higher value of the porosity, the compressibility was found to be the highest [mulberry fibre = 1.76% and aramid = 1.37%] for MF-4 and KV-2. The heat swelling increased with the increasing percentage of mulberry fibre-PAN fibre in the composites [41]. At low (250°C) temperatures, organic fibres produce some hot gases. The 3% polymer composites have shown a minimum value of heat swelling [1.45%] and KV-1 [1.3%]. The density decreased [mulberry fibres-PAN fibre = 2.38–2.14 g/cm^3^ and aramid = 2.45–2.40 g/cm^3^], as their percentage increased in the composition [42]. It might have resulted as mulberry fibre-PAN fibre, and aramid [light in wt.] had replaced the barium sulphate [dense in wt.] in the matrix. A slight difference in values of acetone extraction was observed [mulberry fibre-PAN fibre = 0.59–0.71% and aramid = 0.53–0.57%]. It showed the developed friction materials were properly mixed and cured [43].

It was found that the hardness [HRR] decreases with the increase in mulberry fibre-PAN fibre and aramid in composites [mulberry fibres-PAN fibre = 112.8–103.98 and aramid 116.6–113.22]. The tensile strength was observed to be maximum [mulberry fibres-PAN fibre = 16.8 MPa and aramid = 17.45 MPa] for the MF-2 and KV-1 composites and was the lowest [mulberry fibres-PAN fibre = 15.4 MPa and aramid = 17.34 MPa] for the MF-4 and KV-2. The highest value of tensile modulus [mulberry fibres-PAN fibre = 4050 MPa and aramid = 4213 MPa] was obtained for MF-1 and KV-1, and the lowest value [mulberry fibres-PAN fibre = 3657 MPa and aramid = 4118 MPa] was obtained for MF-4 and KV-2. It indicated that increasing the percentage of mulberry fibres-PAN fibre in the composite leads to a uniform matrix [44]. The impact energy has shown its improved value [mulberry-fibres-PAN fibre = 0.326 J and aramid = 0.289 J] for MF-2 and KV-1, and the lowest value [mulberry fibres-PAN fibre = 0.206 and aramid = 0.276] was observed for MF-4 and KV-2 [45].

### 3.2. Tri-Biological Prosperities of Specimen

The tri-biological prosperities of specimen are described in the following sections.

#### 3.2.1. Response of Friction during Fade Cycles and Recovery Cycles

Table 4 shows the attributes used in tri-biological performance. In the first fade run, it has been found that the Kevlar-based and 3% mulberry fibre-PAN fibre-based composites show the value of *µ* decreases very slowly after reaching the temperature of 220°C, while the other newly developed composites show the value of *µ* falls quickly after reaching the temperature of 150°C [46]. In the second fade cycle, the value of *µ* of Kevlar-based and 3%–6% mulberry fibres-PAN fibre-based composites decreases very slowly after reaching the temperature of 275°C, while the value of *µ* MF-3- and MF-4-based composites decreases very quickly after reaching the temperature of 235°C [47]. In the first recovery cycle, the Kevlar-based and 3%–6% mulberry fibre-PAN fibre-based composites show the value of *µ* increased to 230°C. After that, the value coefficient of friction decreases very slowly, while the MF-3- and MF-4-based composites decrease very fast after reaching the temperature of 160°C [48]. In the second recovery cycle, the Kevlar-based and 3% mulberry fibre-PAN fibre-based composites *µ* values decrease very slowly after reaching the temperature of 260°C. In contrast, other newly developed composites fall quickly after reaching the temperature of 200°C.  Figure 3 shows the developed samples' fade and recovery cycles [49].

#### 3.2.2. Frictional Stability (*Sμ*) and Variability (*Vμ*) Coefficient Behavior

The value of the stability coefficient (*Sμ*) was found to decrease with the increasing percentage of mulberry fibre-PAN and Kevlar in the polymer composite [MF-1 = 0.93, MF-2 = 0.88, MF-3 = 0.84, MF-4 = 0.80, KV-1 = 0.97, and KV-2 = 0.92]. The value of the variability coefficient (*Vμ*) was found to increase with the increasing percentage of mulberry fibre-PAN and Kevlar in the polymer composites [MF-1 = 0.58, MF-2 = 0.60, MF-3 0.63, MF-4 = 0.65, KV-1 = 0.55 and KV-2 = 0.59]. The 3% mulberry fibre-PAN shows the lowest value of variability and the highest stability value.  Figure 4 shows the frictional behavior of S*μ* [stability coefficient] and *Vμ* (variability coefficient) of advanced composites. Polyacrylonitrile is a semi-crystalline organic linear polymer. It has high thermal and mechanical stability and is easily biodegradable. Although it is thermoplastic, it does not melt under normal conditions [50]. The high dipole moment and bulky CN group easily form hydrogen bonds with the copolymers [51].

#### 3.2.3. Fade and Recovery Performance Analysis

During the fade and recovery cycle, it has been noticed that the percentage of fade was found to increase (MF-1 = 32.3, MF-2 = 33.4, MF-3 = 34.3, MF-4 = 36.5, and KV-1 = 30.4 and KV-2 = 32.7) and recovery was also noticed to be increased (MF-1 = 110.6%, MF-2 = 111.9%, MF-3 = 113.8%, and MF-4 = 115.4, KV-1 = 116.8, KV-2 = 116.3) with the increasing percentage of mulberry fibre-PAN and Kevlar in the polymer composites [52].

The reason for increasing the fade and wear percentage with an increased percentage of mulberry fibre-PAN in the polymer composite is that organic fibre develops a heterogeneous matrix and shears easily, acting like third body particles.  Figure 5 shows the frictional behavior of fade %*F* and % *R* of advanced composites [53].

#### 3.2.4. *μP*, *μF*, *μR,* and Δ*μ* Behavior of Composites

During tribological and friction tests, the fluctuation of COF behavior is observed to be increased [MF-1 = 0.220, MF-2 = 0.223, MF = 0.227, MF = 0.231, KV-1 = 0.230, KV-2 = 0.232] and the recovery coefficient is also observed to be increased [MF-1 = .534, MF-2 = 0.558, MF-3 = 0.576, MF-4 = 0.587, KV-1 = .612, and KV-2 = 0.6] as shown in Figure 6, and the performance of COF decreases [MF-1 = 0.35, MF-2 = 0.32, MF = 0.28, MF = 0.26, KV-1 = 0.36, and KV-2 = 0.34], and the fade of COF [MF-1 = 0.548, MF-2 = 0.552, MF = 0.560, MF = 0.566, KV-1 = 0.568, and KV-2 = 0.569] increased with the increase in the mulberry fibre-PAN fibre content in the polymer composites [54]. The motility of perms also decreases due to the excess amount of chromium in the body. Acute tubular and glomerular damage causes higher levels of chromium exposure. The defects in DNA are also increased due to chromium poisoning.

#### 3.2.5. Wear Performance

The wear range for mulberry fibre-PAN composites was between 1.0 and 1.20 g and 0.95–1.05 g for aramid-based polymer composites, as shown in Figure 7. During the wear test, it has been noticed that the wear rate is enhanced with an increased percentage of mulberry fibre-PAN and aramid in composites. MF-1 composite has shown the minimum value of wear, whereas MF-4 has shown the maximum wear value. KV-1 has outperformed KV-2 in terms of results. Some metal processes such as melting, roasting, and extractions are major donors for chromium. Chromium also enters the environment through the daily usage of wood preservatives in chromate copper arsenate (CCA). The increased percentage of mulberry fibre-PAN and aramid fibre in the developed samples does not mix properly with the other ingredients of the polymer composite and increases the wear rate [55].

### 3.3. TGA of Mulberry Fibre-PAN-Based Samples and Kevlar-Based Samples

The TGA was performed on nitrogen and oxygen under two different environmental conditions. It has been noticed that the degradation occurs in three stages for both mulberry-PAN-fibre-based and aramid-based composites. The weight reduction in the first stage has been very low, at less than 13%. In the second stage, a steep or heavy degradation was noticed [56]. The loss was recorded by more than 73%. The third degradation shows the minimum loss in weight. As shown in Figure 8, the first, second, and third degradations were reordered into temperature ranges of 0–240°C, 240–600°C, and 600–900°C, respectively. In a nitrogen environment, the degradation was observed in the temperature ranges of 0–290°C, 290–600°C, and 600–900°C as shown in Figure 8. Heavy losses of more than 76% were observed for the first and third degradations at temperatures ranging from 290 to 600°C, with minimal losses of less than 6% [57]. The first degradation occurs due to the moisture content available in the mulberry fibres-PAN and aramid. The second degradation might be because of the reduction in hydrogen bonding in aramid composites and the loss of hemicelluloses and release of gases from the mulberry fibre-PAN composites [58]. The third degradation occurs due to the loss of the amide group and loss of lignin and cellulose from aramid and mulberry fibre-PAN. This study investigated increasing the mulberry fibre, and aramid percentages in the composites (3–12%) increased the thermal stability [59]. The thermal stability was recorded at a maximum for MF-4. In the case of aramid-based composites, KV-2 shows higher thermal stability [60].

The hydrophilic ionic liquid introduced surface roughness and improved the hydrophilicity of polyacrylonitrile nanofibres. The interlinked nanofibrous structure and the surface chemistry of the nanofibrous membranes are responsible for the higher affinity of the nanofibres for PM2.5 and thus the PM2.5 capture increases for polyacrylonitrile/diethyl ammonium dihydrogen phosphate nanofibre in comparison with polyacrylonitrile nanofibrous membranes [61, 62].

## 4. Conclusions

The following results were evaluated after the end of all physical-chemical, mechanical tribological, and thermal tests:

- The recovery percentage was noticed to be the highest [MF-4 = 115.4 and KV-2 = 116.3] for 12% mulberry-PAN-fibre-based composites. The fade percentage was noticed to be the lowest [MF-1 = 32.3 and KV-1 = 30.4] for 3% mulberry-PAN-fibre-based composites.
- Among all the newly developed samples, 3% mulberry-PAN-fibre-based composites have shown the highest stability coefficient and minimum variability coefficient [stability MF-1 = 0.93 KV-1 = 0.97 and variability = MF-1 = 0.58 KV-1 = 0.55]. The wear was found to be a minimum of 3% for mulberry-PAN-fibre-based composites [MF = 1.0 and KV-1 = 0.95].
- MF-2 [6 wt%] mulberry-PAN-fibre-based brake pad composites have shown better results for ultimate shear strength and proof stress, tensile strength, compressive strength, and impact energy. For 3% mulberry-PAN-fibre-based composites, water absorption, porosity, and compressibility were found to be minimal. The hardness of 3% mulberry-PAN-fibre-based composites was found to be the highest.
- In the comparative study, aramid-based brake pad specimens performed slightly better in %-fade, coefficient of friction, wear performance, and thermal stability than mulberry-PAN fibre-based composites. The performance of the coefficient of friction has shown results for 3% mulberry-PAN-fibre-based composites.
- Thermal stability has shown the highest value of 12 wt. % for mulberry-PAN fibre. Flexural strength, flexural modulus, and tensile modulus show the best performance for 3% brake pad composites among all mulberry-PAN fibre composites.
- The study shows that MF-1 composites show better results for thermal, tri-biological, and mechanical proprieties.

## Figures and Tables

**Figure 1:** (a) PAN fibre. (b) Raw material of mulberry fibre. (c) Developed brake pads of mulberry-PAN fibre.

**Figure 2:** Chase machine for the tribological test.

**Figure 3:** Fade and recovery cycles of developed samples.

**Figure 4:** Frictional Behavior of *Sμ* [stability coefficient] and *Vμ* [variability coefficient] of developed composites.

**Figure 5:** Frictional behavior of fade %*F* and %*R* of developed composites.

**Figure 6:** *µ* Behavior of developed composites.

**Figure 7:** Frictional (COF) and wear behavior of advanced composites.

**Figure 8:** TGA of mulberry-PAN fibre and aramid-based composites in O_2_ and N_2_ atmosphere.

**Table 1:** Composite fabrication details.

Condition for moulding	Procedure
Mixing condition	(i) Proper mixing of basic braking ingredients [phenolic resin, mulberry fibre, PAN fibre/aramid, and Lapinus ingredients for ten minutes]
	(ii) The other remaining ingredients were mixed with previous ingredients [graphite, potassium barium, titane, vermiculite, and aluminum oxide and vermiculite mixed for next another 10 minutes]
Conditions for moulding	*T* = 155°C, pressure (*P*) = 15 MPa, time (*t*) = 10 min,
Condition for oven curing	Time(*t*) = 3 H, *T* = 170°C

where *t* = time, *P* = pressure, *T* = temperature.

**Table 2:** Compositional details of materials.

Fabrication of the composites							
Sr No	Ingredients used	FK-1	FK-2	MF-1	MF-2	MF-3	MF-4
1	Aramid	5	10	0	0	0	0
2	Mulberry fibre [reinforced]	0	0	1.5	3	4.5	6
3	PAN fibre [reinforced]	0	0	1.5	3	4.5	6
4	Alumina [friction]	5	5	5	5	5	5
5	Lapinus [modifier]	15	15	15	15	15	15
6	Potassium titane	5	5	5	5	5	5
7	St. Phenolic Resign [binder] [binder]	10	10	10	10	10	10
8	Graphite [lubricant]	5	5	5	5	5	5
9	Barium [filler]	50	45	52	49	46	43
10	Vermiculite [modifier]	5	5	5	5	5	5

**Table 3:** Characterizations of mulberry fibre and PAN fibre and aramid fibre composites [mechanical, physical, and chemical].

Properties	Standard followed	% and units	3% Kevlar FK-1	6% Kevlar FK-2	3% Fibre [MF-1]	6% Fibre [MF-2]	9% Fibre [MF-3]	12% Fibre [MF-4]
Compressibility	ISO 6310	% [percentage]	1.25	1.37	1.40	1.69	1.73	1.76
Water Absorption	ISO 6310	% [percentage]	1.70	1.80	1.77	1.86	1.90	2.20
Porosity of newly developed composites	JISD 4418 standard	% [percentage]	3.25	3.32	3.4	3.70	4.12	4.05
Heat swelling	SAE J 160 JNU80	% [percentage]	1.3	1.76	1.45	1.53	1.74	1.79
Ash content	ASTMD570-98	% [percentage]	75.30	72.48	74.75	74.07	72.98	71.06
Density	ASTM C271/C271 M-16	(g/cm3) [Gram per centimeter cubic]	2.45	2.40	2.38		2.20	2.14
Hardness	Rockwell-R-scale	HRR	116.6	113.2	112.8	111.6	109.5	103.9
Acetone extraction	ASTMD494	% [percentage]	0.57	0.53	0.59	0.64	0.68	0.71
Impact energy	Standard	(J) [joule]	0.289	0.276	0.252	0.326	0.224	0.206
Shear strength	ASTM D256	(kgf) [kilogram force]	1870	2090	2267	2520	1932	1721
Tensile strength	ASTM D732	(MPa) [Mega-Pascal]	17.45	17.34	15.4	16.8	13.2	11.8
Flexural strength	ASTM E8	(MPa) [Mega-Pascal]	62.83	60.23	59.78	55.37	51.12	50.34
Tensile modulus	ASTM D790	(MPa) [mega-Pascal]	4450	4518	4257	3956	3784	3657
Flexural modulus	ASTM E8	(GPa) [Mega-Pascal]	2.60	2.78	2.55	2.50	2.35	2.30
Failure strain	ASTM D790	(%) [Percentage]	1.20	1.24	1.48	1.54	1.60	1.69
Proof stress	ASTM E8	(MPa) [Mega-Pascal]	3.4	2.9	2.8	3.6	3.2	2.75
Ultimate compressive strength	ASTM E8	(MPa) [Mega-Pascal]	162.3	167.5	165.7	176 7	160.9	140.6

**Table 4:** Attributes used in Tri-biological performance.

Attributes used	Favourable
Wear rate	Wear should show minimum values
COP	Coefficient performance should show the highest values
Recovery%	Recovery percentage should be high as possible and favourable more than 100%
% Fade	Fade should show minimum values
*µ*R	The recovery coefficient should show the highest values
*µ*v	The variability coefficient should show the lowest values
∆*µ*	The fluctuation coefficient should show minimum values

## Data Availability

The data used to support the findings of this study are included within the article. Further data or information can be obtained from the corresponding author upon request.
